# On Fatigue Detection for Air Traffic Controllers Based on Fuzzy Fusion of Multiple Features

**DOI:** 10.1155/2022/4911005

**Published:** 2022-10-11

**Authors:** Yi Hu, Zhuo Liu, Aiqin Hou, Chase Wu, Wenbin Wei, Yanjun Wang, Min Liu

**Affiliations:** ^1^College of Civil Aviation, Nanjing University of Aeronautics and Astronautics, Nanjing, Jiangsu 210016, China; ^2^School of Information Science and Technology, Northwest University, Xi'an, Shaanxi 710127, China; ^3^Department of Data Science, New Jersey Institute of Technology, Newark, NJ 07102, USA; ^4^Department of Aviation and Technology, San Jose State University, San Jose, CA 95192, USA; ^5^Zhongke Haoyin Intelligent Technology Co., Ltd., Hefei, Anhui 230088, China

## Abstract

Fatigue detection for air traffic controllers is an important yet challenging problem in aviation safety research. Most of the existing methods for this problem are based on facial features. In this paper, we propose an ensemble learning model that combines both facial features and voice features and design a fatigue detection method through multifeature fusion, referred to as Facial and Voice Stacking (FV-Stacking). Specifically, for facial features, we first use OpenCV and Dlib libraries to extract mouth and eye areas and then employ a combination of M-Convolutional Neural Network (M-CNN) and E-Convolutional Neural Network (E-CNN) to determine the state of mouth and eye closure based on five features, i.e., blinking times, average blinking time, average blinking interval, Percentage of Eyelid Closure over the Pupil over Time (PERCLOS), and Frequency of Open Mouth (FOM). For voice features, we extract the Mel-Frequency Cepstral Coefficients (MFCC) features of speech. Such facial features and voice features are fused through a carefully designed stacking model for fatigue detection. Real-life experiments are conducted on 14 air traffic controllers in Southwest Air Traffic Management Bureau of Civil Aviation of China. The results show that the proposed FV-Stacking method achieves a detection accuracy of 97%, while the best accuracy achieved by a single model is 92% and the best accuracy achieved by the state-of-the-art detection methods is 88%.

## 1. Introduction

The 2006-2015 statistics of flight incidents in China broken down by causes show that human factors account for 25.67% [1]. From 1994 to 2020, there are 97 accidents in China caused by air traffic controllers [2]. Also, a survey on controller fatigue from National Transportation Safety Board (NTSB) shows that a number of major investigations identify fatigue as a probable cause, contributing factor, or a finding [3]. The above studies and statistics have made it very clear that timely and accurate fatigue detection for air traffic controllers performing control and command operations on site is critical to minimizing aviation safety hazards. Fatigue detection is mainly divided into subjective detection and objective detection. Subjective detection is to classify and quantify the fatigue status based on the subject's subjective performance. The detection methods in this category have the advantages of convenient operation and low cost, and have been widely adopted. However, they also suffer from some disadvantages such as poor real-time performance and the impact of human subjective consciousness. Subjective detection methods can be further divided into three subcategories: questionnaires and subjective evaluation forms, oral question-and-answer analysis, and active detection models. Lee and Kim developed hypotheses and survey questions based on interviews with 929 pilots and conducted a nationwide survey. They concluded that inadequate planning operation, flight direction, culturally different partnership, aircraft environment, job assignment, racial difference, hotel environment, and other factors can cause pilot fatigue [4]. Jiang et al. designed a questionnaire based on Theory of Planned Behavior (TPB), which effectively reveals the psychological factors related to fatigue driving [5].

Objective detection has the advantages of high accuracy and reliability, and it is not affected by the subject's subjective consciousness. The methods in this category have become the focus of research for fatigue detection and can be divided into the following two subcategories: contact and noncontact. Most traditional contact-based methods for fatigue detection measure physiological signals such as electrocardiograms and brain waves [6, 7]. Such methods through body contact are able to yield high detection accuracy but may interfere with the normal operation of air traffic controllers. Most noncontact-based methods mainly track facial expressions, such as mouth state detection [8], eye tracking [9, 10], and reaction time [11]. Verma et al. proposed to detect fatigue by comparing the location of the joints of the current posture [12]. Since noncontact methods are noninvasive and easy to instrument, they have received a great deal of attention.

In this paper, we propose a fatigue detection method through multifeature fusion based on ensemble learning, referred to as Facial and Voice Stacking (FV-Stacking). Specifically, for facial features, we first use OpenCV and Dlib libraries to extract mouth and eye areas and then employ a combination of M-Convolutional Neural Network (M-CNN) and E-Convolutional Neural Network (E-CNN) to determine the state of mouth and eye closure based on five features, i.e., blinking times, average blinking time, average blinking interval, Percentage of Eyelid Closure over the Pupil over Time (PERCLOS), and Frequency of Open Mouth (FOM). For voice features, we extract the Mel-Frequency Cepstral Coefficients (MFCC) features of speech. Such facial features and voice features are fused using a carefully designed stacking model for fatigue detection. The stacking framework increases the amount of information used for ensemble learning and can integrate different types of features by choosing and stacking appropriate base models. Real-life experiments are conducted on 14 air traffic controllers in Southwest Air Traffic Management Bureau of Civil Aviation of China. The experimental results show that the proposed FV-Stacking method achieves a detection accuracy of 97%, while the best accuracy achieved by a single model is 92%, and the best accuracy achieved by the state-of-the-art detection methods is 88%. The main contributions of our work are summarized as follows:

1. We develop a machine learning model that can recognize the closed state of the mouth and eyes with high accuracy
2. We fuse speech features and facial features to detect the fatigue state of air traffic controllers
3. We design an FV-Stacking ensemble learning model and achieve an accuracy rate of 97% for fatigue detection

The rest of this paper is organized as follows.  Section 2 conducts a survey of related work.  Section 3 details the design of the proposed ensemble learning model through multifeature fusion.  Section 4 presents and analyzes experimental results. We conclude our work in Section 5.

## 2. Related Work

Fatigue detection is used in various scenarios and is mainly divided into two categories, i.e., subjective detection and objective detection.

In subjective methods, fatigue ranges are often used. Williamson et al. [13] systematically studied the impact of lack of sleep on fatigue and established a set of subjective methods that can be used to assess fatigue. De Vries et al. [14] claimed that the Fatigue Assessment Scale is the most promising fatigue measure, where workers are requested to fill out questionnaires before and after work to divide the fatigue scale.

Among objective methods, there are contact methods and noncontact methods for fatigue detection, depending on whether or not the testing tool needs to physically touch the tested person during testing. Heart rates, brain waves, and electrocardiograms (EEG) are often used as common indicators in contact-based detection methods. Arnau et al. [15] used EEG to study the relationship between mental fatigue and age. Murugan et al. [7] extracts 13 electrocardiogram (ECG) signal features and classifies them through machine learning to determine the fatigue status of a person. Chen et al. [16] determined whether or not the air traffic controller is fatigued by measuring physiological information including flicker fusion threshold, thumb/index finger strength, and systolic and diastolic pressure before and after work. For noncontact detection, many methods consider facial expressions and voice signals. Dinges and Grace [17] proposed PERCLOS, a physical quantity measuring fatigue/drowsiness, which is defined as a certain percentage (e.g., 70% or 80%) of time when the eyes are closed per unit time. Generally, a tested person is considered to be fatigued if PERCLOS exceeds a certain threshold. Zhang et al. [18] used a convolutional neural network to determine the closure status of eyes, calculated PERCLOS based on this, and combined the number of blinks per unit time to identify the fatigue state. Nie et al. [19] used PERCLOS, blink rate, and eye closure time to detect fatigue status. Gu et al. [20] detected fatigue status by calculating PERCLOS and yawn frequency. Similarly, voice features are also considered in some noncontact methods for fatigue detection. Shen et al. [21] used Revised Fractal Dimension Feature to determine the fatigue status of air traffic controllers.

## 3. Ensemble Learning Thorough Multifeature Fusion

Ensemble learning accomplishes the learning task by combining multiple models. The selection of an ensemble learning model follows the principle of “good but different”. It uses a series of base models and some rules to integrate multiple learning results to obtain a final one, which is expected to outperform a single learning method [22]. Ensemble learning includes several schemes, these are Bagging, Stacking, Boosting, Blending, etc.

We propose a model of FV-Stacking to combine facial features and voice features for fatigue detection. Stacking is a layered model integration framework. The first layer is composed of multiple base learners. In the FV-Stacking framework, we combine five base models, i.e., Logistic Regression (LR), Decision Tree (DT), Support Vector Machine (SVM), Long Short-Term Memory (LSTM), and Convolutional Neural Network (CNN), which take the original training dataset as input. The second layer is a simple LR model, which takes the output of the base learners in the first layer as input. The architecture of the proposed FV-Stacking framework is shown in Figure 1.

A brief introduction to each of the base models used in FV-Stacking is provided as follows.

1. *LR*. Logistic regression uses the logistic function sigmoid to map the result of linear regression to the range of [0,1]. In FV-Stacking, LR is used in both the first and the second layers. In the first layer, logistic regression classifies fatigue status based on facial features, while in the second layer, it is used to classify the combined inputs of all base models
2. *SVM*. Support vector machine is a classification model, and its basic model is a linear classifier with the largest interval defined in the feature space. The key idea is to solve the separating hyperplane that can correctly divide the training dataset and have the largest geometric interval. In this paper, we use a linear support vector machine to recognize facial features
3. *DT*. Decision tree is a supervised machine learning algorithm based on a tree structure, in which each internal node represents a judgement of an attribute, each branch represents the result of a judgement, and each leaf node represents a classification method. In this paper, we use CART decision tree to recognize facial features
4. *LSTM*. Long Short-Term Memory is a recurrent neural network and is well-suited to classify time series data. In this paper, LSTM is used to process MFCC features, as illustrated in Figure 2

(5) *CNN*. Convolutional neural network is a type of neural network that performs convolution calculation and has a deep structure. It includes multiple layers including convolutional layer, pooling layer, and fully connected layer. The convolutional layer and the pooling layer perform feature extraction on the input data, and the fully connected layer performs a nonlinear combination of the extracted features to obtain the output. In this paper, CNN is used to process MFCC features, using three convolutional layers, three pooling layers, a flatten operation, one fully connected layer, and one sigmoid classifier, as illustrated in Figure 3

The input of FV-Stacking includes visual data and voice data. The facial feature input includes blinking times, average blinking time, average blinking interval, PERCLOS, and FOM. The voice feature input is the MFCC feature.

### 3.1. Facial Feature Extraction

#### 3.1.1. Face Detection and Feature Point Extraction

Face detection is to determine face images, and feature point extraction is to identify feature points in face images. These are the most critical steps in facial recognition. The quality of a detected face and the accuracy of the feature point location directly affect the results of subsequent processes. In this paper, we use Dlib Library to detect faces and extract facial feature points. Dlib is a modern C++ toolkit that includes a variety of machine learning algorithms and tools, providing high-quality machine learning, image processing, deep learning, and face recognition library [23]. Face recognition algorithms include face detection, face feature extraction, and face feature vector calculation. Hence, we choose the Dlib library to implement a high-quality face recognition system. In the Dlib library, the pretrained facial landmark detector is used to estimate the location of 68 coordinates (*x*, *y*) that map to facial structures on the face. For illustration, the indexes of the 68 coordinates are visualized in Figure 4. In this paper, we employ the Dlib library to extract the 68 coordinates of the face and locate the eye and the mouth.

#### 3.1.2. Eye Closure Status Recognition

After extracting 68 eye detection points, we use these points to construct an eye area of size 32 × 26 based on the facial landmarks defined in Eq. (1), as illustrated in Figure 5.  Figure 5(a) is the marked points of a human eye in the video, and Figure 5(b) is the extracted grayscale image of the human eye.

(1) $$\begin{array}{c} w_{e}=1.2*X,\\ H_{e}=\frac{w_{e}*34}{26}. \end{array}$$

Once the eye area is identified, we use E-CNN to determine the eye's closure status [24]. E-CNN contains three convolutional layers, three pool layers, two fully connected layers, a flatten operation, and one sigmoid classifier, as illustrated in Figure 6 [25]. The input is a grayscale image of size 26 × 34 × 1.

#### 3.1.3. Mouth Closure Status Recognition

Among 68 facial detection points, we use those points of mouth to extract the mouth area of size 120 × 80, based on the facial landmarks defined in Eq. (2). An extraction result is plotted in Figure 7 for illustration.  Figure 7(a) is the marked points of an air traffic controller's mouth in the video, and Figure 7(b) is the extracted grayscale image of the air traffic controller's mouth.

(2) $$\begin{array}{c} W_{m}=1.2*Y_{m},\\ H_{m}=\frac{w_{m}*120}{80}. \end{array}$$

Once the mouth area is identified, we use M-CNN to determine the mouth's closure status [26]. Convolutional neural networks contain three convolutional layers, three pool layers, two fully connected layers, a flatten operation, and one sigmoid classifier, as illustrated in Figure 8.

The input is a grayscale image of size 80 × 120 × 1.

#### 3.1.4. Eye and Mouth Features

We generated two queues when identifying air traffic controllers in the video stream with M-CNN and E-CNN. As shown in Figure 9, the first queue stores the detection results of eye state, and the second queue stores the detection results of mouth state. We use a flag number to represent the closure state of the eye or mouth in each frame: the flag ‘1' indicates that the eye or mouth is open, and the flag ‘0' indicates that the eye or mouth is closed.  Figure 9(a) is a queue that stores the closure state of the mouth with M-CNN, and Figure 9(b) is a queue that stores the closure state of the eye with E-CNN.

We derive five features of eye and mouth from the queues, i.e., blinks, average blinking time, average blink time interval, PERCLOS, and FOM, as defined below:

1. *Blinks*. The number of blinks is measured over a fixed time period. As the level of fatigue increases, the number would also change
2. *Average Blinking Time (ABT)*. It measures the average number of eye closures per blink in a fixed time period, which is often related to fatigue, calculated as

(3) $$\begin{array}{c} \text{ABT}=\frac{n_{\text{close}}}{N_{\text{blinks}}}, \end{array}$$

where *n*_close_ is the total number of eye-closed frames, and *N*_blinks_ is the total number of blinks over a period of time.

(3) *Average blink time interval (ABTI)*. *t* refers to the average empty time intervals in a fixed time period, calculated as

(4) $$\begin{array}{c} \text{ABTI}=\frac{\sum_{\text{i}=\text{n}}^{\text{n}}{\text{t}}_{\text{interval}}}{{\text{N}}_{\text{blinks}}-1}, \end{array}$$

where *n* denotes the number of blink time intervals, and *t*_interval_ denotes the single blink time interval.

(4) *PERCLOS*. The ratio between the number of frames with closed eyes and the total number of frames in unit time, calculated as

(5) $$\begin{array}{c} \text{PERCLOS}=\frac{n_{\text{close}}}{N_{\text{total}}}, \end{array}$$

where *n* denotes the number of frames with closed eyes and *N* denotes the total number of frames.

(5) *FOM*. Similar to PERCLOS, it refers to the ratio between the number of frames with closed mouth and the total number of frames in unit time, calculated as

(6) $$\begin{array}{c} \text{FOM}=\frac{n_{\text{closedmouth}}}{N_{\text{total}}}, \end{array}$$

where *n*_closedmouth_ denotes the number of frames with closed mouth and *N*_total_ denotes the total number of frames

### 3.2. Vocal Feature Extraction

It is critical to extract the most representative voice signal features for fatigue detection. In this paper, we employ MFCC feature extraction from voice signals as this unique cepstrum-based extraction method is more in line with the principle of human hearing, and it is also the most common and effective speech feature extraction algorithm. The MFCC extraction process is illustrated in Figure 10.

As shown in Figure 10, MFCC consists of seven steps, each of which has its own function and mathematical approach as discussed briefly below:

1. *Preemphasis*. Preemphasis is a filtering method that emphasizes higher frequencies to balance the spectrum of voiced sounds that have a steep roll-off in the high-frequency region
2. *Framing*. To facilitate speech analysis, voice signal can be divided into small segments, which are referred to as frames. Each frame contains *N* sampling points in an observation unit. Typically, *N* is set to be 256 or 512, and the time covered is about 20-30 ms
3. *Windowing*. Voice is constantly changing in a long range and cannot be processed without fixed characteristics. Therefore, each frame is substituted into a window function, and the value outside the window is set to be 0. Commonly used window functions include square window, Hamming window, and Hanning window, etc. Considering the characteristics of a window function in the frequency domain, Hamming window is often used
4. *Discrete Fourier Transform (DFT)*. Each windowed frame is converted into magnitude spectrum by applying DFT, calculated as

(7) $$\begin{array}{c} X\left(k\right)=\overset{N-1}{\underset{i=0}{\sum }}x\left(n\right)e^{\left(-j2\pi nk\right)/N},\;0\leq K\leq N-1, \end{array}$$

where *N* is the number of points used to compute the DFT

(5) *Mel Spectrum*. Mel spectrum is computed by passing the Fourier transformed signal through a set of band-pass filters known as Mel-filter bank. The Mel scale is approximately a linear frequency spacing below 1 kHz and a logarithmic spacing above 1 kHz. The approximation of Mel from physical frequency is calculated as

(8) $$\begin{array}{c} f_{\text{Mel}}=2569\log_{10}\left(1+\frac{f}{100}\right), \end{array}$$

where *f* denotes the physical frequency in Hz, and *f*_Mel_ denotes the perceived frequency

(6) *Discrete Cosine Transform (DCT)*. DCT is applied to the transformed Mel frequency coefficients to produce a set of cepstral coefficients
(7) *Dynamic MFCC features*. Cepstral coefficients are usually referred to as static features, since they only contain information from a given frame. The extra information about the temporal dynamics of the signal is obtained by computing the first and second derivatives of cepstral coefficients

## 4. Experiments and Performance Evaluation

### 4.1. Experimental Platform

In this work, we use OpenCV [27] and Dlib libraries to process video dataset and use Keras and Sklearn frameworks to construct the model for fatigue detection. The entire detection system is implemented and tested on a Windows 10 PC equipped with 32GB of memory and a GPU with 8GB memory.

### 4.2. Dataset

For E-CNN, we collect 8,598 images with eyes open and 6,510 images with eyes closed. Altogether, we use 12,086 eye images for training and 3,022 images for testing. Similarly, for M-CNN, we collect 2,155 images with mouth open and 1,980 images with mouth closed. Altogether, we use 3,721 mouth images for training and 414 images for testing.

We also collect video and audio data of air traffic controllers in real operation. We collect 14,673 video and audio clips, where the length of each video is 15 seconds and the length of each audio is 7 seconds. Accordingly, we obtained 14,673 facial features and MFCC features from such video and audio data, out of which 11,738 are used for training the proposed FV-Stacking ensemble learning model, and 2,935 are used for testing.

### 4.3. Experiments

For the video data, we use OpenCV and Dlib to extract the eyes and mouth of each air traffic controller in each video frame, and then we use E-CNN and M-CNN models to identify the state of the eyes and mouth. Finally, five features are calculated, including blinks, average blinking time, average blink time interval, PERCLOS, and FOM. For the audio data, we obtained an MFCC feature vector of size 20 × 244 through the MFCC feature extraction process.

The facial features (i.e., blink times, average blinking time, average blink time interval, PERCLOS, and FOM) and MFCC features extracted from the audio are passed to the ensemble learning model as input. We use FV-Stacking to combine facial features and MFCC features to determine whether or not the air traffic controller is fatigued. The overall detection process is illustrated in Figure 11.

### 4.4. Experimental Results and Analysis

To verify the classification performance of M-CNN, ECNN, and FV-Stacking, we consider recall rate, precision, accuracy, *f*_1_ score, and AUC (Area Under Curve) as the main performance metrics in our experiments, as defined in the following:

1. Recall

(9) $$\begin{array}{c} \text{recall}=\frac{\text{TP}}{\text{TP}+\text{FN}}, \end{array}$$

where TP and FN denote the number of true positives and the number of false-negatives, respectively. This metric represents the proportion of positive samples that are correctly identified as a percentage of the total positive samples

(2) Precision

(10) $$\begin{array}{c} \text{precision}=\frac{\text{TP}}{\text{TP}+\text{FN}}, \end{array}$$

where FP denotes the number of false-positives. This metric represents the portion of correctly identified positive samples as a percentage of all samples that are identified as positive

(3) Accuracy

(11) $$\begin{array}{c} \text{accuracy}=\frac{\text{TN}+\text{TP}}{\text{TN}+\text{TP}+\text{FP}+\text{FN}}, \end{array}$$

where TN denotes the number of true negatives. This metric represents the proportion of correctly classified samples to the total number of samples

(4) *f*_1_ score

(12) $$\begin{array}{c} f_{1}=\frac{2\cdot \text{recall}\cdot \text{precision}}{\text{recall}+\text{precision}} \end{array}$$

This metric is based on the harmonic average of the recall rate and the precision rate.

(5) *Area Under Curve (AUC)*. A schematic diagram of the ROC (Receiver Operating Characteristic) curve is plotted in Figure 12. The horizontal axis of the curve is the false positive rate, calculated as

(13) $$\begin{array}{c} \text{FPR}=\frac{\text{FP}}{\text{TN}+\text{FP}}, \end{array}$$

while the vertical axis is the true positive rate, calculated as

(14) $$\begin{array}{c} \text{TPR}=\frac{\text{TP}}{\text{TP}+\text{FN}}. \end{array}$$

In Figure 12, the area under the ROC curve and the horizontal axis is defined as the Area Under Curve (AUC). Obviously, the value of this area is no greater than 1. Moreover, because the ROC curve is generally above the line *y* = *x*, the value range of AUC is between 0.5 and 1. The closer the AUC is to 1.0, the better performance the detection method achieves.

The performance of E-CNN and M-CNN is shown in Table 1.

To evaluate the performance of FV-Stacking, we compare and analyze the recall rate, precision, accuracy, *f*_1_ score, and AUC of single models and FV-Stacking. The results are plotted in Figure 13.

From Figure 13, we observe that the best recall rate of signal models is 90%, the precision is 92%, the accuracy is 90%, the *f*_1_ score is 90%, and the AUC is 0.96. The recall of FV-Stacking proposed in this paper reaches 97%, the precision reaches 97%, the accuracy reaches 97%, the *f*_1_ score reaches 97%, and the AUC reaches 0.99. These results show that FV-Stacking consistently outperforms any single model.

In some other methods, different features are used for fatigue detection. For example, in the work by Zhang et al. [18], fatigue is judged by PERCLOS and blinking frequency. In the work by Nie et al. [19], fatigue is judged by blink time, PERCLOS, blinks, and blink frequency. In the work by Gu et al. [20], fatigue is judged by PERCLOS and FOM. One common strategy is to determine the fatigue state by setting fixed thresholds for different characteristics. For example, in the work by Zhang et al. [18], the PERCLOS threshold is set to be 0.25, and in the work by Nie et al. [19], the PERCLOS threshold is set to be 0.06. In [20], Gu et al. set the PERCLOS threshold to be 0.5. However, in different scenarios, such fixed thresholds may not always yield the best performance. In order to mitigate the impact of thresholds on the performance, we combine different features using various machine learning models including Support Vector Machine (SVM), K-Nearest Neighbor (KNN), and Logistic Regression (LR) to compare the performance of different fatigue detection methods, as summarized in Table 2.

From Table 2, we observe that the best recall rate of different fatigue detection methods is 89%, the accuracy is 88%, the *f*_1_ score is 88%, the precision is 89%, and the AUC is 0.93. The recall rate of the proposed FV-Stacking method reaches 97%, the accuracy reaches 97%, the *f*_1_ score reaches 97%, the precision reaches 97%, and the AUC reaches 0.99. These results show that FV-Stacking consistently outperforms other fatigue detection methods.

## 5. Conclusion and Future Direction

Civil aviation aircraft has become an indispensable tool for our daily travel. Route management at airports is becoming increasingly complicated as the airport size and the aircraft volume continue to grow. Such intensive work leads to fatigue of air traffic controllers, which is one of the major factors for accidents.

We focused on the fatigue detection problem for air traffic controllers. To improve detection accuracy, we combined facial features including blinks, average blink duration, average blink interval, PERCLOS, and yawn frequency as well as the MFCC characteristics of voice signal. We designed an ensemble learning method for fatigue detection and used real-life video and audio data for performance evaluation.

This research has resulted in the following findings:

1. Both M-CNN and E-CNN are able to accurately identify the open and closed state of the mouth and eyes
2. By strategically combining facial and speech features, the proposed ensemble learning model, FV-Stacking, is able to achieve consistently better detection performance in comparison with single models and other detection methods, in terms of various performance metrics

Our work provides a new perspective for the development of fatigue detection methods by combining facial features and vocal features. The proposed approach achieves a high fatigue detection rate and has a great potential to effectively avoid accidents caused by the fatigue of air traffic controllers.

There are many alternative vocal features in addition to MFCC. It is of our future interest to experiment with other vocal features such as Single Frequency Filtering Cepstral Coefficients (SFFCC) [28, 29] and Zero-Time Windowing Cepstral Coefficients [30]. Moreover, we plan to incorporate some other features that may also reflect the fatigue state of air traffic controllers, such as sitting posture [12].

## Figures and Tables

**Figure 1:** FV-Stacking architecture.

**Figure 2:** LSTM structure.

**Figure 3:** CNN structure.

**Figure 4:** The location of 68 feature points on a face.

**Figure 5:** Eye identification.

**Figure 6:** E-CNN structure.

**Figure 7:** Mouth identification.

**Figure 8:** M-CNN structure.

**Figure 9:** The process for obtaining the closure state of the mouth and eyes.

**Figure 10:** MFCC feature extraction.

**Figure 11:** A schematic block diagram.

**Figure 12:** AUC based on ROC.

**Figure 13:** Performance comparison between different models.

**Table 1:** the performance of CNN.

Model	Recall	Precision	Accuracy	*f*_1_ score	AUC
E-CNN	98%	98%	98%	98%	0.99
M-CNN	97%	98%	97%	97%	0.99

**Table 2:** Performance comparison between different methods.

	Our method	Work by Zhang et al. [18]			Work by Nie et al. [19]			Work by Gu et al. [20]		
		LR	SVM	KNN	LR	SVM	KNN	LR	SVM	KNN
Precision	97%	85%	85%	88%	85%	86%	89%	0.83%	85%	73%
Accuracy	97%	84%	84%	88%	85%	85%	88%	82%	82%	71%
Recall	97%	86%	86%	89%	85%	85%	89%	83%	85%	70%
*f*_1_ score	97%	85%	85%	88%	85%	85%	89%	83%	83%	70%
AUC	0.99	0.93	0.93	0.92	0.93	0.93	0.92	0.91	0.91	0.83

## Data Availability

The data used in this paper is not public. We have signed a confidentiality agreement with Southwest Air Traffic Management Bureau of Civil Aviation of China because these facial videos and voices were collected from the air traffic controllers performing tasks in the real environment in the Management Bureau of Civil Aviation.
